This article has been retracted.

# Investigation and Countermeasures on Mental Health Status of Applied Fresh Graduates from the Perspective of Psychological Capital

**DOI:** 10.1155/2022/5352958

**Published:** 2022-09-28

**Authors:** Yuanzhen Zeng

**Affiliations:** Mental Health Education and Consultation Center, Guangxi Agricultural Vocational and Technical University, Nanning, 530001 Guangxi, China

## Abstract

Based on the perspective of psychological capital, the mental health status of applied college graduates is analyzed, and the corresponding countermeasures are put forward. Questionnaires are issued to investigate the mental health status of fresh graduates. The BSSI score of male students (102.05 ± 2.01) is not significantly different from that of female students (*P* > 0.05). SCL-90 scores of male students include somatization (1.95 ± 0.01), compulsion (1.84 ± 0.15), interpersonal relationship (1.75 ± 0.14), depression (1.92 ± 0.08), anxiety (1.70 ± 0.10), hostility (7.25 ± 0.16), terror (1.35 ± 0.41), bigotry (1.29 ± 0.17), and psychosis (1.33 ± 0.64). There is no significant difference compared with those of female students (*P* > 0.05). SCL-90 scores of high stress graduates include somatization (2.00 ± 0.17), compulsion (2.30 ± 0.08), interpersonal relationship (1.61 ± 0.20), depression (1.87 ± 0.09), anxiety (1.80 ± 0.11), hostility (1.30 ± 0.20), terror (1.39 ± 0.14), paranoid (1.48 ± 0.10), and psychosis (1.50 ± 0.11). There is significant difference between forced and low pressure graduates (*P* < 0.05). There is no statistical significance in other items (*P* > 0.05). Colleges and universities need to work together with fresh graduates to deal with negative emotions and stress, so as to improve mental health and promote employment.

## 1. Introduction

The experts led by Luthans and others believed that psychological capital was “a positive psychological state displayed by individuals in the process of growth and development, specifically manifested as self-efficacy, optimism, hope and resilience.” Psychological capital referred to in the research includes the following four dimensions.

Self-efficacy (Figure 1) refers to people's belief that they can complete a certain task or work behavior [1]. It involves not the skill itself, but the degree of confidence that one can use the skill to complete the behavior [2]. Self-efficacy is an individual's degree of self-determination and trust. It is a kind of belief. A person's self-efficacy is not related to his actual ability or skill but has a great influence on his behavior. People with a strong sense of self-efficacy are confident in dealing with problems when facing adverse situations. They are willing to accept challenges and make efforts in a strange and changing environment. They believe that they can change difficulties and are more likely to achieve goals. However, people with low self-efficacy lack confidence in themselves. They are more likely to retreat, be anxious, and be restless when facing pressure and difficulties and are prone to have escape psychology and avoidance behaviors, which are not conducive to achieving goals [3, 4].

Professor Selingman, an American psychologist, used attributive styles to distinguish optimism from pessimism [5]. In his opinion, optimism refers to that individuals make their own, lasting, and universal attributions to positive events while making external, temporary, and specific attributions related to the situation to negative events when interpreting the events that have occurred. In the face of difficulties, setbacks, and failures, optimistic people can regard misfortune or change as an opportunity and challenge. They can face with a positive attitude and see the potential of all kinds of opportunities. In the pursuit of difficult goals, optimistic people can persevere unremittingly. They have positive expectations for the future and keep making efforts, with a belief that they will eventually achieve success.

Kim, S. H. defined hope as a positive motivational state formed on the basis of the experience generated by the interaction between the motivation for success (the energy of targeted feedback) and the path (plan to achieve the goal). Hope is a positive state of individual motivation. A person who is hopeful about the future sets challenging goals based on the realities of himself and his environment and finds ways to achieve his personal goals through perseverance. Hopeful people take the initiative to set goals in life and try to solve problems effectively [6]. They have the ability of independent thinking and will achieve their goals through active rather than passive waiting and gradually achieve their goals through their own positive attitude, unremitting efforts, and various methods. The targeted feedback is shown in Figure 2.

Resilience refers to an individual's ability to persevere, maintain confidence, quickly recover from happiness, and find ways to achieve success when faced with difficulties or adversity. It is an important factor for an individual to overcome hardship, walk out of adversity, and march towards success. It is also known as resilience and mental resilience. People with high resilience can actively deal with difficult problems when they are in trouble, make themselves stronger and more flexible in failure and adversity, and quickly recover their psychological state and even reach a better state. In challenging positive events, individuals with high resilience can develop their potential abilities with extraordinary willpower to help individuals eventually get out of difficulties [7].

## 2. Literature Review

### 2.1. Psychological Capital

Improving psychological capital is beneficial to the career development of college students. College students are facing the transformation from students to social and professional people and facing a series of conflicts and contradictions from the society, family, and their own growth. Whether they can grow up healthily, the play of many abilities is affected by psychological capital. College students who have a strong sense of self-efficacy are strong, optimistic, and full of hope for the future and are better able to adapt to the society and the workplace [8]. On the contrary, it is prone to psychological problems and occupational maladjustment, which may lead to insurmountable obstacles and even a vicious circle in the future personal career development. If college students can have more psychological capital, possess optimistic and confident psychological quality, and be full of hope for the future, they can deal with various problems better in life. In this way, in the development of his or her career (Figure 3), he or she can “respond to all changes with the same changes,” which will benefit him or her immensely [9].

Accumulating psychological capital is beneficial to cultivating innovative and entrepreneurial talents. In August 2012, the General Office of the Ministry of Education issued a document requiring entrepreneurship courses to be offered in regular colleges and universities across the country. The move is intended to promote the all-round development of college students and speed up the process of building China into a power of human resources. At present, China's entrepreneurship education is in its infancy, and many college students lack confidence, correct self-recognition, practical experience, and ability to solve practical problems. They are full of hope and confused about the future. In study and life, there is a lack of real role models and realistic goals to strive for. It is difficult to carry out innovation and entrepreneurship education in such student groups. Because of this, it is particularly important to develop the psychological capital of college students, and it is extremely urgent to carry out entrepreneurship education in colleges and universities. On the one hand, entrepreneurship education can awaken and excavate the psychological capital of college students. On the other hand, psychological capital of college students can be accumulated and improved (Figure 4) [10, 11].

Increasing psychological capital is helpful to improve the employability of college students. The rise of psychological capital theory provides a new perspective for improving the job-hunting competitiveness of college students [12]. With abundant psychological capital, college students are more likely to succeed in their first employment and become more comfortable in their future career development. Many college students cannot find a job because of their poor ability and low quality, and employability cannot meet the requirements of employers. Ability and personality become the focus of employers' investigation. Employers want applicants to have self-management ability, unity and cooperation ability, interpersonal communication ability, initiative learning ability, and creative problem-solving ability. Employers prefer candidates with positive attitude, confidence and thirst for knowledge, honest words and actions, and ability to work under pressure (Figure 5) [13]. The self-introduction, leaderless group discussion, psychological test, and other links in the process of interview and written examination all examine the ability and personality of college students from different angles.

Paying attention to psychological capital is beneficial to realize its synergistic effect with human capital and social capital. In recent years, the joint effect of human capital, social capital, and psychological capital on college students' job hunting and personal career has attracted the attention of human resource managers in universities, college students, and enterprises. Human capital includes individual education, certificates, training experience, and knowledge experience. Social capital refers to the network of social relationships in which an individual is a member and can utilize them. Psychological capital includes positive psychological qualities such as self-confidence, optimism, resilience, and hope. Three-dimensional capital is indispensable in the development of individual career. These three aspects transform and influence each other and finally make individuals obtain a perfect career. Some college students devote themselves to study only for scholarships and certificates, hardly taking part in any extracurricular activities. Some university student cadre, because of the work reason and organizing all kinds of activities, often play truant and fail frequently. Some college students are mediocre in academic performance and have no self-established social relationship network (Figure 6). They do not know how to turn to others for help when they encounter problems [14, 15].

### 2.2. Mental Health of College Students

Mental health is very important for a person. It means that a person's physiology, psychology, and society are in a harmonious state with each other. Its characteristics are as follows.

Normal intelligence (Figure 7): this is the most basic psychological condition for people's life, study, work, and labor [16].

Emotional stability and happiness: this is an important sign of mental health. It shows that a person's central nervous system is in relative balance, meaning that the body functions in harmony. A mentally healthy person's behavior is coordinated, his behavior is controlled by consciousness, his thought and behavior are coordinated, and he has the ability to control himself. If a person's behavior and thought contradict each other, his attention is not focused, his thoughts are confused, his language is fragmented, and his work is chaotic. Psychological adjustment should be carried out.

Good interpersonal relationship (Figure 8): living in society, one should be good at getting along with others, help others, and establish good interpersonal relationship. People's communication activities can reflect people's mental health state. Normal friendly communication between people is not only a necessary condition to maintain mental health but also an important method to obtain mental health [17].

Good adaptability: living in a complicated and changeable world, people will encounter a variety of environments and changes in their life. Therefore, a person should have good adaptability. No matter realistic how the environment has changed, one will be able to get used to the mental health. A person's mental health is not necessarily in every aspect of performance. As long as in life practice, he can correctly understand himself.

Sound will: will is a psychological process of choosing, deciding, and performing a purposeful activity. The one with sound will shows a higher level in the action of the consciousness, decisiveness, tenacity and self-control, and other aspects. Students with sound will have a conscious purpose in all kinds of activities. They can make timely decisions and use a practical and prepared way to solve the problems encountered. In the face of difficulties and setbacks, they can take a reasonable way of reaction and can control emotions in action and words and deeds.

Complete personality (Figure 9) [18, 19]: personality refers to the sum total of the individual's relatively stable psychological characteristics. Perfect personality refers to a sound and unified personality, that is, what an individual thinks, says, and does is coordinated and consistent. One is the integrity and unity of all elements of personality structure, such as having correct self-consciousness, not producing self-identity mix, taking positive and enterprising outlook on life as the core of personality, and taking this as the center of their own, needs, goals, and actions together.

Correct self-evaluation: correct self-evaluation is the important condition of college students' mental health. College students perform self-observation, self-recognition, self-judgment, and self-assessment, so as to achieve self-knowledge and appropriately know themselves. They can accept themselves, with self-esteem, self-improvement, self-control, and moderate self-love. They can face up to the reality. With the reform of the cultural system and the proposal of the national slogan of “education for all,” the number of new college students in our country is increasing. With the increasing number of college students, the mental health problems of college students are becoming more and more serious.

### 2.3. Psychology of Fresh Graduates

With the reform of China's economic structure and system, the problem of difficult employment of college students has become more prominent, and the psychological problems of college students have aroused widespread social concern. Since the expansion of college entrance examination in 1999 (Figure 10), college education has turned from elite education to mass education, with the enrollment growth rate of ordinary colleges and universities reaching 42%, the average annual growth rate of college enrollment reaching 30%, and the enrollment rate exceeding 60% [20].

College students are no longer popular. Employment pressure and emotional problems have become the main psychological problems of fresh graduates. On the one hand, colleges and universities need to take various measures to promote employment and, at the same time, need to carry out employment psychological counseling through multiple channels. Anxiety is the basic emotion developed by college students in the process of struggling with the changing situation and adapting to the survival. Moderate anxiety can fully mobilize the function of each organ and improve the reaction speed and alertness of individual brain. According to the survey, anxiety is the main psychological problem of fresh college students, who are worried about the changing environment and the transformation of social roles. Maintaining a moderate level of anxiety can create stress. Anxiety is a normal psychological reaction. This moderate psychological pressure, to some extent, is to urge themselves, which can stimulate college students' enterprising spirit, so as to participate in the employment competition more actively. It manifests itself as being self-motivated and enterprising. With graduation time is coming, the vast majority of students are anxious. They should learn to talk. Talking out is an important method in psychological counseling. If you feel anxious during the employment process, please try to talk to your classmates, friends, and family, and seek the help of a professional psychologist. For the college graduates' psychological counseling work, universities should pay attention to the emotional guidance, such as guiding students to understand and vent their own emotions. Setbacks are inevitable. Individuals should learn to motivate themselves and carry out positive self-suggestion, such as maintaining an optimistic and confident psychological state. They should reduce the negative impact of adverse psychological factors and maintain a healthy psychological state [21].

Blind following psychology refers to a psychological phenomenon in which individuals abandon their original ideas and opinions and adopt conformity due to the influence or pressure of group behavior in communication. It is a social psychological phenomenon prevalent in university campuses. The social causes of blind following are complex. College students lack the consciousness of making personal career planning. They are out of touch with the society and unable to fully understand the needs of the social industry. They lack in-depth professional learning, social practice experience, and decision-making ability. Therefore, under the influence of the herd mentality, when choosing a career, they tend to follow what others say and go with the flow, lack of a comprehensive analysis of their own ability, and lack of due decisiveness and persistence when making decisions. Blind following psychology not only hinders college students to play their own subjective initiative but also limits the potential of college students to play in a deeper level. They are easy to lose themselves and unable to overcome their own limitations to achieve greater achievements. To avoid the bind following psychology, fresh graduates need to be personalized when making career plans. That is, according to their own conditions and requirements, combined with professional development prospects and social development interests, a rational employment plan with personalized characteristics is formulated. They also need to know their own interests, temperament, and personality. Rational thinking is conducive to the development of a full-life career. They should adjust career mentality and correct understanding of self. Self-development is very important [22].

## 3. Methods

### 3.1. Research Object

Under the premise of voluntary participation, a total of 359 medical students from 8 classes in a medical university were selected as the object of the questionnaire survey. Finally, 325 valid questionnaires were collected with a recovery rate of 90.53%. There were 143 male graduates aged 23-25 with an average age of 23.55 (SD, 0.70) years and 182 female graduates aged 23-24 with an average age of 23.19 (SD, 0.35) years. All the graduates involved in the survey have completed the undergraduate study and can be awarded the bachelor's degree according to the regulations of the university [23].

### 3.2. Survey Methods

1. General investigation: a preliminary investigation and statistics were made on the gender, age, success of postgraduate entrance examination (admission notice shall prevail), and employment (employment agreement shall prevail) of the graduates who participated in the survey
2. Beck Pressure Scale was used to measure the stress status of medical college graduates. Beck-Srivastava Stress Inventory (BSSI) consisted of 46 items, which could be used to investigate the stressors and stress intensity of graduates. In terms of pressure sources, 6 items were designed and the graduates were asked to rank the most common items such as economic pressure, love pressure, interpersonal relationship, family problems, academic problems, prospects, and employment, so as to determine the most important pressure sources faced by the graduates. In terms of stress intensity, 40 items were designed and each item was scored on a scale of 1-5, with 1 indicating “no pressure,” 2 indicating “very light pressure,” 3 indicating “moderate pressure,” 4 indicating “excessive pressure,” and 5 indicating “great pressure.” Four factors closely related to stress intensity, including learning pressure (specifically associated with 10 items), economic pressure (specifically associated with 10 items), interpersonal relationship (specifically associated with 10 items), and clinical practice (specifically associated with 10 items), can be tested and scored. The scores of specific associated items of each factor were added to obtain the total score of the factor, and the total scores of the four factors were added to obtain the final BSSI score. According to the standards set by the original work, the detection criteria of graduates with great pressure are as follows.

(1) $$\begin{array}{c} \text{BSSI Factor score}\geq 3\text{ score},\\ \text{BSSI Total score}\geq 72\text{ score} \end{array}$$

Cronbach's *a* of BSSI was confirmed by using it in premedical students and domestic adolescents as follows.

(2) $$\begin{array}{c} \text{BSSI}=0.82∼0.90. \end{array}$$

Therefore, it can accurately detect the pressure of graduates who participate in the survey.

Symptom Check List 90 (SCL-90), also known as the symptom self-rating scale, consists of 90 items. Each item is scored on a 1-5 scale, with 1 indicating “no symptoms,” 2 indicating “very mild symptoms,” 3 indicating “moderate symptoms,” 4 indicating “severe symptoms,” and 5 indicating “severe symptoms.” Somatization (12 items of specific association), compulsion (10 items of specific association), interpersonal relationship (9 items of specific association), depression (13 items of specific association), anxiety (10 items of specific association), hostility (specific association six items), horror concrete association (7 items of specific association), paranoid (6 items of specific association), and psychosis (7 items of specific association) closely related to mental health factors are tested (another 7 items without specific factor, in as “other”). The total score of the associated items of each factor is added to obtain the total score of the factor, and the total score of the 10 factors is added to obtain the final SCL-90 score. The detection criteria for possible mental health problems are as follows.

(3) $$\begin{array}{c} \text{SCL}-90\text{Total score}\geq 160\text{score},\\ \text{Positive factor number}\geq 43\text{item},\\ \text{The average of a single factor points}\geq 2\text{score}. \end{array}$$

Cronbach's *α* of SCL-90 in domestic medical students can reach 0.945, so it can accurately detect the mental health status of graduates involved in the survey.

(3) Quality control

The whole process of the survey was completed under the guidance of student management workers (counselors or deputy secretaries of the General Branch of the CPC, all with national psychological counseling teacher qualification). If the graduates who participated in the survey have any questions about the specific questions of the questionnaire, they are answered on the spot. Incomplete answers, difficult to identify after alteration, and L ≥ 7 points in TABP questionnaire were excluded.

(4) Statistical treatment

All inputs were recorded by statistical professionals and processed by SPSS20.0 statistical analysis software. If the quantitative variables followed normal distribution, mean ± standard deviation (*X* ± SD) was used to describe them; otherwise, median (interquartile spacing) was used to represent them. On the premise that the relevant quantitative variables approximately conform to the normal distribution, multiple linear regression was used to analyze the specific factors affecting the mental health of medical college graduates. For the comparison of quantitative data between the two groups, *t* test was used if the variance was uniform; otherwise, rank sum test was used, and *P* < 0.05 was used as the criterion for statistically significant difference.

## 4. Results

### 4.1. Mental Health Status Score

The BSSI score of male students (102.05 ± 2.01) shows no statistical significance compared with that of female students (*P* > 0.05), as shown in Table 1.

### 4.2. Mental Health Status by Gender

SCL-90 scores of male students include somatization (1.95 ± 0.01), compulsion (1.84 ± 0.15), interpersonal relationship (1.75 ± 0.14), depression (1.92 ± 0.08), anxiety (1.70 ± 0.10), hostility (7.25 ± 0.16), terror (1.35 ± 0.41), bigotry (1.29 ± 0.17), and psychosis (1.33 ± 0.64) which had no significant difference compared with female students (*P* > 0.05). See Table 2.

### 4.3. Mental Health Status of Different Mental Capital

SCL-90 scores of high stress graduates include somatization (2.00 ± 0.17), compulsion (2.30 ± 0.08), interpersonal relationship (1.61 ± 0.20), depression (1.87 ± 0.09), anxiety (1.80 ± 0.11), hostility (1.30 ± 0.20), terror (1.39 ± 0.14), paranoid (1.48 ± 0.10), and psychosis (1.50 ± 0.11). There is significant difference between forced and low pressure graduates (*P* < 0.05). There is no statistical significance for other items (*P* > 0.05), as shown in Table 3.

## 5. Conclusions

Developing and accumulating psychological capital of college students is the bounden responsibility of universities and college students themselves. The psychological capital of college students can be fully explored only when universities and students make joint efforts to create a good atmosphere and conditions and make full use of the environment and resources in all aspects.

### 5.1. Campus Environment

The school needs to create a harmonious and loose campus culture environment, improve the psychological quality of students, and cultivate the soil for the growth of college students' psychological capital. The campus culture can improve college students' sense of identity and belonging and encourage them to read, study, practice, and participate in various activities of enthusiasm, initiative, and creativity. Through a variety of promotions, management system, and evaluation system, colleges and universities should promote and encourage all students to participate in various campus culture activities and practice, so as to find and focus on a few college students with no practical experience. For this part of the students, the psychological capital is scarce. They are in urgent need to be provided psychological assistance. College mental health education and counseling center should intensify propaganda, build a set of mature psychological problem prevention and intervention mechanism through a variety of forms, and make college students actively seek counseling staff to help when meeting problems, so as to ensure that the college students' psychological problems can be found in time and more serious problems can be avoided.

### 5.2. Career Guidance

Colleges and universities should improve the employment guidance work, pay attention to the rich resources of college students, and improve the students' self-confidence. Colleges and universities should improve the employment guidance institutions, ensure that the division of labor is clear, enhance the service consciousness of staff, and highlight their professionalism. The employment guidance institutions of colleges and universities should maintain cooperation with professional talent assessment, intermediary agencies, and employers. The employment guidance should run through college students' career planning, job hunting guidance, entrepreneurship education, and follow-up investigation after entry. College students' own resources should be explored and utilized through the personal achievement stories, career interviews, and career experience reports, so as to encourage each other, experience success repeatedly, and enhance the sense of self-efficacy. Through students to tell about the positive qualities of self-confidence, sincerity, diligence, tenacity, optimism, and gratitude of people and things, multilevel model groups are established, so as to improve the value system of college students and enhance the confidence of college students to enter the society and employment.

### 5.3. Social Support

College students should be pleased with themselves, actively engage in practice, establish their own social support system, and develop and improve their psychological capital. Many college students cannot recognize their own advantages, nor can they face up to or even try to cover up their shortcomings. They are unable to accept and be pleased with themselves, and it is difficult to produce real confidence. Only when college students tolerate and accept everything about themselves, cherish the present, plan the future carefully, and believe that their imperfect selves can still create a wonderful life can they truly possess self-confidence. College students can accumulate experience, improve their knowledge structure, improve practical ability, and cultivate innovative spirit by actively participating in various extracurricular practical activities. Lack of social practice and work experience is an important reason for many college students' employment difficulties. A college student who actively participates in social practice shows maturity, self-confidence, optimism, and active communication and coordination skills. Therefore, when encountering various difficulties in life, study, and emotion, he or she can be more patient and actively try to solve problems. An effective social support system can give college students confidence and strength when they encounter setbacks, so that they can recover their courage and have a strong will and finally overcome difficulties and achieve success. The psychological capital stored by college students will extend to their future professional life and long-term life development. Therefore, colleges and universities should fully realize the importance of developing the psychological capital of college students, create a good campus environment, and provide necessary support for college students, so as to realize the educational function of the university. College students themselves should be deeply aware of the important role of psychological capital in promoting employability and career development and continue to accumulate their own positive psychological capital, improve their competitiveness, and take responsibility for their own development.

## Figures and Tables

**Figure 1:** Self-efficacy.

**Figure 2:** Targeted feedback.

**Figure 3:** Career planning.

**Figure 4:** Causes of low psychological capital of college students.

**Figure 5:** Employment of college students.

**Figure 6:** Social network.

**Figure 7:** Intelligence of college students.

**Figure 8:** Harmonious interpersonal relationship.

**Figure 9:** Classical personality composition.

**Figure 10:** College entrance examination expansion.

**Table 1:** Mental health status score.

Gender	Male students	Female students	*P*
BSSI score	102.05 ± 2.01	94.51 ± 1.05	<0.05

**Table 2:** Mental health status by gender.

SCL-90	Male students	Female students	*P*
Somatization	1.95 ± 0.01	1.94 ± 0.02	>0.05
Compulsion	1.84 ± 0.15	1.87 ± 0.09	>0.05
Interpersonal relationship	1.75 ± 0.14	1.74 ± 0.10	>0.05
Depression	1.92 ± 0.08	2.00 ± 0.10	>0.05
Anxiety	1.70 ± 0.10	1.71 ± 0.20	>0.05
Hostility	7.25 ± 0.16	7.31 ± 0.04	>0.05
Terror	1.35 ± 0.41	1.40 ± 0.02	>0.05
Paranoid	1.29 ± 0.17	1.30 ± 0.10	>0.05
Psychosis	1.33 ± 0.64	1.34 ± 0.58	>0.05

**Table 3:** Mental health status of different mental capital.

SCL-90	High pressure	Low pressure	*P*
Somatization	2.00 ± 0.17	1.99 ± 0.10	>0.05
Compulsion	2.30 ± 0.08	1.80 ± 0.11	<0.05
Interpersonal relationship	1.61 ± 0.20	1.60 ± 0.09	>0.05
Depression	1.87 ± 0.09	1.87 ± 0.15	>0.05
Anxiety	1.80 ± 0.11	1.74 ± 0.19	>0.05
Hostility	1.30 ± 0.20	1.31 ± 0.15	>0.05
Terror	1.39 ± 0.14	1.40 ± 0.13	>0.05
Paranoid	1.48 ± 0.10	1.45 ± 0.20	>0.05
Psychosis	1.50 ± 0.11	1.47 ± 0.12	>0.05

## Data Availability

The labeled data set used to support the findings of this study is available from the corresponding author upon request.
